# Manta Ray Foraging Optimization with Vector Quantization Based Microarray Image Compression Technique

This article has been retracted.

**DOI:** 10.1155/2022/7140552

**Published:** 2022-05-25

**Authors:** Nora A. Alkhaldi, Rawabi Abdulaziz Abdullah Alsedais, Hanan T. Halawani, Sayed M. Abdelkhalek Aboutaleb

**Affiliations:** ^1^Department of Computer Science, College of Computer Sciences and Information Technology, King Faisal University, Al Ahsa 31982, Saudi Arabia; ^2^Department of Computer Science, College of Computer Science and Information Systems, Najran University, Najran 61441, Saudi Arabia; ^3^Department of Mathematics, Faculty of Science, Sohag University, Sohag 82524, Egypt

## Abstract

DNA microarray technologies enable the analysis of the expression of numerous genes in an individual experiment and become an important approach in the field of medicine and biology for investing genetic function, regulation, and interaction. Microarray images can be investigated well for obtaining the contained genetic data. But is it undesirable to retain the genetic data and avoid the microarray images? Due to considerable attention to DNA microarray and several experiments being performed under distinct conditions, a massive quantity of data gets produced over the globe. In order to store and share the microarray images, effective storage and communication models are needed in a natural way. Vector quantization (VQ) is a commonly utilized tool for compressing images, which mainly aims to produce effective codebooks comprising a collection of codewords. Therefore, this paper presents a manta ray foraging optimization (MRFO) with Linde–Buzo–Gray (LBG) based microarray image compression (MRFOLBG-MIC) technique. The LBG model is commonly utilized to design local optimal codebooks to compress images. The construction of codebooks can be defined as a nondeterministic polynomial time (NP) hard problem and can be resolved by the MRFO algorithm. The codebooks produced from LBG-VQ are optimized using the MRFO algorithm to attain optimum optimal codebooks. When the codebooks are produced by the MRFOLBG-MIC algorithm, Deflate model can be applied to compress the index tables. The design of the MRFO algorithm with LBG and Deflate based index table compression demonstrate the novelty of the work. For demonstrating the enhanced compression efficacy of the MRFOLBG-MIC model, a wide-ranging experimental validation process is performed using a benchmark dataset. The experimental outcomes inferred that the MRFOLBG-MIC model accomplished superior outcomes over the other existing models.

## 1. Introduction

Microarray analysis is a mechanism that permits the evaluation and categorization of genes in the fastest means. Currently, a microarray is considered the foremost tool for gene-related investigation [1]. The microarray technique is utilized for monitoring a huge amount of tissue array images in a simultaneous way. All microarray experiment generates many larger-sized images that become difficult to share or store [2]. Such an enormous number of microarray images implies new challenges for bandwidth resources and memory space. Lacking high speed Internet connection, it is hard or not possible to distribute microarray images from some other parts of the world [3]. Various researches were carried out for handling the memory of a huge number of microarray image datasets effectively. The image compression method is one of the means for handling such a greater amount of images. Generally, the main motive of the image compression technique is sending an image with fewer bits [4, 5].

Image compression has three elements, namely, realization of unwanted data in image, transformation method, and suitable coding method [6]. The most significant image compression standard is JPEG and its quantization is classified into two kinds such as vector quantization (VQ) and scalar quantization (SQ). It is an inconvertible compression technique and is widely utilized in the compressing of images, which includes some loss of information [7]. The main motive of VQ is producing an optimum codeword (CW) which comprises a collection of CWs, where else an input image vector is allotted on the basis of minimal Euclidean distance. The familiar VQ method is Linde–Buzo–Gray (LBG) model. LBG technique provides flexibility, simplicity, and adaptability. Moreover, the technique relies on lower Euclidean distance amongst respective CWs and image vectors. It could produce local optimal solutions and in other words, it had failed in presenting the best global solutions. The final solution of the LBG algorithm depends on an arbitrarily-created codebook at the early stages.

The VQ method was utilized for few more years. Historically, VQ was detached into 3 stages: vector decoding, vector encoding, and codebook generation. The generation of the codebook is the most significant function, which determines the efficiency of VQ [8]. The motive of codebook generation is identifying code vector (codebook) for provided sets of training vectors by reducing the average pairwise distance among the training vectors and their respective CWs. The vector encrypting operation of VQ methods comprises the partition of the image into more input vectors (or blocks), and then a comparison is made to the CWs of the codebook with a view to identifying the nearest CW for every input vector [9]. The VQ encodes each and every input vector towards an index of the codebook. Generally, the codebook size is comparatively very small with actual image data sets, and thus the intention of image compression is attained. In the decoding process, the connected subimages are accurately recovered by the encoded codebook. When each and every subimage is entirely recreated, the decoding is finished. The codebook model of the VQ algorithm was done by most of the researchers [10].

Codebook training can be treated as a challenging process in VQ due to the fact that the codebook significantly influences image compression quality. The importance of codebook training process has received significant attention among research communities to design evolutionary optimization algorithms such as monarch butterfly optimization (MBO) [11], slime mould algorithm (SMA) [12], moth search algorithm (MSA) [13], hunger games search (HGS) [14], Runge Kutta method (RUN) [15], colony predation algorithm (CPA) [16], weIghted meaN oF vectOrs (INFO) [17], mayfly optimization [18], Harris hawks optimization (HHO) [19], and Manta ray foraging optimization [20]. In this study, the MRFO algorithm is used over other metaheuristics due to its simplicity, easy to implement, highly versatile, few adjustable parameters, and flexibility.

This paper presents a manta ray foraging optimization (MRFO) with Linde–Buzo–Gray (LBG) based microarray image compression (MRFOLBG-MIC) technique. Primarily, the LBG model is commonly utilized to design local optimal codebooks to compress images. By the use of VQ, the local codebooks are produced to reduce the mean square error (MSE) and increase the peak signal to noise ratio (PSNR). The codebooks produced from LBG-VQ are optimized using the MRFO algorithm to attain optimum optimal codebooks. Therefore, the output image received is reconstructed with the enhanced codebooks obtained by the proposed model for microarray image compression. This optimal compression algorithm produces efficient codebooks by generating visually better-quality images. When the codebooks are produced by the MRFOLBG-MIC algorithm, Deflate model can be applied to compress the index tables. For ensuring the improved compression efficacy of the MRFOLBG-MIC model, a wide-ranging experimental validation process is performed using a benchmark dataset.

## 2. Related Works

The authors in [21] implemented a novel technique taking benefit of the potential simplicity of the run length technique for contributing a volumetric RLE method for binary medicinal information from the 3-D procedure. The presented volumetric-RLE (VRLE) technique varies in the 2-D RLE method employing correlations of intraslice only that is utilized to compressing binary medicinal information employing voxel-correlation of interslice. Geetha et al. [22] presented a VQ codebook construction technique named as L2-LBG approach employing the Lempel–Ziv–Markov chain algorithm (LZMA) and Lion optimization algorithm (LOA). If the LOA created the codebook, LZMA was executed for compressing the index table and higher the compression performance of LOA. Kumar et al. [23] execute the LBG with BAT optimized technique that creates a suitable codebook. An optimized technique was utilized not only for the codebook proposal along with for the codebook size chosen.

In [24], the application of bat optimized technique in medicinal image compression was identified. The bat optimized technique was utilized here to optimal codebook design from Vector Quantization (VQ) technique. The efficiency of the BAT-VQ compression model has been related to the recent approaches. Kumari et al. [25] presented the flower pollination algorithm (FPA) based vector quantization to optimum image compression with optimum reconstructed image quality. The performances of the presented approach were estimated by utilizing mean square error (MSE), fitness function (FF), and peak signal to noise ratio (PSNR). In [26], the whale optimization algorithm (WOA) was utilized for determining an optimum codebook from image compression. In WOA, there are distinct searching approaches, and it is an ideal technique to find an optimum codebook from image compression. Execution of the presented technique to compression on many typical images illustrates that the presented approach compresses images with suitable quality.

Othman et al. [27] examined a novel effectual lossy image compression approach dependent upon the polynomial curve fitting approximation approach that signifies several pixels of the image with less amount of polynomial coefficients. The projected approach begins with changing the image to a 1D signal and it separates this 1D signal into segments of variable length. Afterward, the polynomial curve fitting was executed for these segments for constructing the coefficient matrix. In [28–31], ML techniques are trained for relating the clinical image content to its compression ratio. When trained, the optimal DCT compression ratio of X-ray images was selected on offering an image to networks. The experimental outcomes demonstrated that the radial basis function neural network (RBFNN) learning technique is effectually utilized for classifying the optimal compression ratio to the X-ray image but maintained superior image quality.

## 3. The Proposed Model

In this work, a new MRFOLBF-MIC model is presented to compress microarray images for effective storage and transmission. The LBG model is commonly utilized to design local optimal codebooks to compress images. The construction of codebooks can be defined as a nondeterministic polynomial time (NP) hard problem and can be resolved by the MRFO algorithm. When the codebooks are produced by the MRFOLBG-MIC algorithm, Deflate model can be applied to compress the index tables.

### 3.1. Overview of VQ

VQ is resolved as a block coding method deployed to compressed images with loss data. In VQ, the codebook structure is a vital procedure [32]. Assuming *Y*={*y*_*ij*_} represents the raw image size of M × M pixels that are separated into discrete block sizes of n × n pixels. Specifically, an input vector *X*=(*x*_*i*_, *i*=1,2,…, *N*_*b*_) comprises a group of *N*_*b*_=[*N*/*n*] × [*N*/*n*] and L represents n × n. An input vector *x*_*i*_, *x*_*i*_ ∈ *ℜ*^*L*^ is *L* dimension Euclidean spaces. The codebook C has *L* dimensionality codewords, in which *C*={*c*_1_, *c*_2_,…, *c*_*N*_*c*__}, *c*_*j*_ ∈ *ℜ*^*L*^, ∀*j*=1,2,…, *N*_*c*_. Each input vector has represented by a row vector *x*_*i*_=(*x*_*i*_1, *x*_*i*2_,…,  *x*_*iL*_) and the j^th^ codeword of the codebook was implied as *c*_*j*_=(*c*_*j*1_, *c*_*j*2_,…, *c*_*jL*_). An optimized C by means of MSE that enhances the minimized distortion function D. Commonly, the lesser value of *D* represented optimum C.

(1) $$\begin{array}{c} D\left(C\right)=\frac{1}{N_{b}}\sum_{j=1}^{N_{c}}\sum_{i=1}^{N_{b}}\mu_{ij}\cdot {\left\|x_{i}-c_{j}\right\|}^{2}. \end{array}$$

Subject to the constraint provided in the following equations:.

(2) $$\begin{array}{c} \sum_{j=1}^{N_{c}}\mu_{ij}=1,\forall i\in \left\{1,2,\ldots ,N_{b}\right\}, \end{array}$$

(3) $$\begin{array}{c} \mu_{ij}=\left\{\begin{array}{c} 1\text{if}x_{i}\text{isinthejthcluster,}\\ 0. \end{array}\right.\; \end{array}$$

And, *L*_*k*_ ≤ *C*_*jk*_ ≤ *U*_*k*_, *k*=1,2,…, *L*, where *L*_*k* _ implies the lesser k^th^ component from trained is a vector and *U*_*k*_ demonstrates the superior k^th^ component from the input vector. The ‖*x*_*i*_ − *c*_*i*_‖ illustrates Euclidean distance among the vector x and CW c.

### 3.2. Process Involved in LBQ

The LBG is demonstrated as a scalar quantization approach founded by Lloyd in the year 1957 and it can be generalized to VQ from the year 1980. It uses 2 existing states for input vectors for determining the codebook. Assume *x*_*i*_, *i*=1,2,…, *N*_*b*_ refers to the input vector, distance function *d*, and initial codewords *c*_*j*_(0), *j*=1,2,…*N*_*c*_ in Figure 1 demonstrates the steps in LBG. The LBG technique frequently employed 2 states for achieving optimally codebook dependent upon the provided methods [32]:

(i) Split the input vector into distinct groups utilizing minimal distance rules. The resultant block was stored in *N*_*b*_ × *N*_*c*_ binary indicator matrix U in which the components are demonstrated as follows:
  (4) $$\begin{array}{c} \mu_{ij}=\left\{\begin{array}{cc} 1, & \text{if}d\left(x_{i},c_{j}\left(k\right)\right)=\underset{p}{\text{min}}d\left(x_{i},c_{p}\left(k\right)\right),\\ 0, & \text{otherwise.} \end{array}\right. \end{array}$$
(ii) Distinguish the centroid of each portion. The preceding codewords are exchanged by some accessible centroids.
  (5) $$\begin{array}{c} c_{j}\left(k+1\right)=\frac{\sum_{i=1}^{N_{b}}\mu_{ij}\cdot x_{i}}{\sum_{i=1}^{N_{b}}\mu_{ij}}. \end{array}$$
(iii) Go to step 1 if there are still no alterations in *c*_*j*_ happening.

### 3.3. Codebook Construction Using MRFO Algorithm

In this work, the construction of codebooks can be defined as an NP hard problem and can be resolved by the MRFO algorithm. MRFO has been evolved by 3 foraging natures, namely, cyclone, somersault, and chain foraging. The arithmetical methods are defined in the following [33].

### 3.4. Chain Foraging

In MRFO, MR has the capacity to observe the position of plankton and move towards them. Once the position of plankton is high, it is taken as an optimal one. Even though the best solution is dark room, MRFO considers the optimum solution as plankton with higher MR would reach the best food source. An individual without first moving towards food is not operated; however, it has emerged from them. Hence, an individual is upgraded by an optimal solution that is identified in front of it. The mathematical method of chain foraging is expressed as follows:

(6) $$\begin{array}{c} x_{i}^{d}\left(t+1\right)=\left\{\left.\begin{array}{c} x_{i}^{d}\left(t\right)+r\cdot \left(x_{\text{best}}^{d}\left(t\right)-x_{i}^{d}\left(t\right)\right)+\alpha \cdot \left(x_{\text{best}}^{d}\left(t\right)-x_{i}^{d}\left(t\right)\right)i=1,\\ x_{i}^{d}\left(t\right)+r\cdot \left(x_{i-1}^{d}\left(t\right)-x_{i}^{d}\left(t\right)\right)+\alpha \cdot \left(x_{\text{best}}^{d}\left(t\right)-x_{i}^{d}\left(t\right)\right)i=2,\ldots ,N, \end{array}\right.\right.\;\\ \alpha =2\cdot r\cdot \sqrt{\left|\text{log}\left(r\right)\right|}\;. \end{array}$$

Here, *r* indicates an arbitrary number within [0,1]*a* symbolizes a weight coefficient, *x*_*i*_^*d*^(*t*) represents the location of *i* th individual at time *t* in *dt*  *h* dimension, and *x*_best_^*d*^(*t*) refers to the plankton with higher concentration. The position upgrade of *ith*  individual can be represented by the location *x*_*i*−1_(*t*) of the (*i* − 1)th individual along with location *x*_best_(*t*) of the food.

### 3.5. Cyclone Foraging

Once a group of MR finds dense plankton in marine water, it increases the long foraging chain and moves to the food in a spiral path. Like spiral foraging principles that are recognized in WOA. In the cyclone foraging technique of MR, spiral motion for MR swim in front of it. Also, follow a point in front of it and move toward food in a spiral manner. It can be arithmetically expressed as follows:

(7) $$\begin{array}{c} \left\{\begin{array}{c} X_{j}\left(t+1\right)=X_{\text{best}}+r\cdot \left(X_{i-1}\left(t\right)-X_{i}\left(t\right)\right)+e^{bw}\cdot \text{cos}\left(2\pi w\right)\cdot \left(X_{\text{best}}-X_{i}\left(t\right)\right),\\ Y_{i}\left(t+1\right)=Y_{\text{best}}+r\cdot \left(Y_{i-1}\left(t\right)-Y_{i}\left(t\right)\right)+e^{bw}\cdot \text{sin}\left(2\pi w\right)\cdot \left(Y_{\text{best}}-Y_{i}\left(t\right)\right). \end{array}\right. \end{array}$$

Here, *w* denotes an arbitrary value within [0,1], *X*_best_ and *Y*_best_ represent the food with the highest concentration. The motion behaviour is transmitted to *n*‐D space. The numerical approach to cyclone foraging is illustrated by the following equation:

(8) $$\begin{array}{c} x_{i}^{d}\left(t+1\right)=\left\{\begin{array}{c} x_{\text{best}}^{d}+r\cdot \left(x_{\text{best}}^{d}\left(t\right)-x_{i}^{d}\left(t\right)\right)+\beta \cdot \left(x_{\text{best}}^{d}\left(t\right)-x_{i}^{d}\left(t\right)\right)i=1,\\ x_{\text{best}}^{d}+r\cdot \left(x_{i-1}^{d}\left(t\right)-x_{i}^{d}\left(t\right)\right)+\beta \cdot \left(x_{\text{best}}^{d}\left(t\right)-x_{i}^{d}\left(t\right)\right)i=2,\ldots ,N, \end{array}\right.\\ \beta =2e^{r_{1}T-t+1/T}\cdot \text{sin}\left(2\pi r_{1}\right), \end{array}$$

where *β* denotes the weight coefficient, *T* characterizes a large amount of iterations, and *r*_1_ indicates rand value within [0,1].

The individual implements an exploration in terms of food as the position; thus the cyclone foraging has the best exploitations for a region with an optimum solution. As well, it is implied for improving the search procedures. It highly concentrates on searching technique and activates MRFO to obtain the extreme global search is represented as follows:

(9) $$\begin{array}{c} x_{\text{rand}}^{d}=Lb^{d}+r\cdot \left(Ub^{d}-Lb^{d}\right),\\ x_{i}^{d}\left(t+1\right)=\left\{\begin{array}{c} x_{\text{rand}}^{d}+r\cdot \left(x_{\text{rand}}^{d}-x_{i}^{d}\left(t\right)\right)+\beta \cdot \left(x_{\text{rand}}^{d}-x_{i}^{d}\left(t\right)\right)i=1,\\ x_{\text{rand}}^{d}+r\cdot \left(x_{i-l}^{d}\left(t\right)-x_{i}^{d}\left(t\right)\right)+\beta \cdot \left(x_{\text{rand}}^{d}-x_{i}^{d}\left(t\right)\right)i=2,\ldots ,N. \end{array}\right.\; \end{array}$$

Now *x*_rand_^*d*^ indicates the arbitrary position that is produced from searching space, *Lb*^*d*^ and *Ub*^*d*^ denotes lower and upper bounds.  Figure 2 illustrates the flowchart of the MRFO technique.

### 3.6. Somersault Foraging

In this process, the position of food is specified as an important factor. Consequently, it upgrades the locations around an optimum location. It can be arithmetically expressed as follows:

(10) $$\begin{array}{c} x_{i}^{d}\left(t+1\right)=x_{i}^{d}\left(t\right)+S\cdot \left(r_{2}\cdot x_{best}^{d}-r_{3}\cdot x_{i}^{d}\left(t\right)\right),i=1,\ldots ,N. \end{array}$$

Now *S* signifies the somersault factor that chooses somersault rank, and *S*=2, *r*_2_, and *r*_3_ indicate arbitrary value within [0, 1].  It is possible for a person to swim towards the position for seeking an application situated among symmetrical and existing locations. The distance amongst a better and individual location is minimized, and the perturbation of the existing position is reduced. The individual can be explored by the best solution in a searching space. The pseudocode of the MRFO algorithm is given in Algorithm 1.

An input image can be separated into a nonoverlapping block that endures quantization by the LBG method. The codebook that is utilized utilizing the LBG method was trained with the MRFO technique that is for satisfying requires of global convergence and declaring global convergence. The index numbers are sent on the broadcast medium and recreated at target utilizing the decoded. The transformed index and equivalent codewords were set correctly for the drive of creating decompressed image size nearly equivalent to providing an input image.

**Step 1 .**

*Initialized Parameters*: at this point, the codebook created utilizing the LBG method was stated that the primary solution whereas residual solutions were established in an arbitrary approach. The reached solution signifies the codebook of *N*_c_ codewords.

**Step 2 .**

*Choosing the Current Optimum Solution*: the fitness of all solutions are procedure and select the superior fitness place as the better outcome.

**Step 3 .**

*Creating New Solution*: the place of manta rays is upgraded by utilizing the prey place. If the arbitrarily produced number (K) is superior to ∼a, afterward exchange the bad places with the recently identified position and keep an optimally place unchanged.

**Step 4 .**

Rank the solution in the application of fitness function (FF) and select an optimal solution.

**Step 5 .**

*End Condition*: by Following the steps 2 and 3 still obtaining the termination criteria.

### 3.7. Codebook Compression Process

Once the codebooks are created by the MRFOLBG-MIC algorithm, Deflate model can be used to compress the index tables. It comprises a sequence of blocks indicating succeeding blocks of input data. Every individual block can be coded by the integration of the LZ77 model and Huffman coding. The first LZ77 model identifies recurrent substrings and substitutes them with backward reference. It utilizes a reference to a duplicated string that exists in the identical or earlier blocks up to 32K input bytes back. It is utilized in gzip, an extended version of LZ77. It mainly determines the repeated strings in the input data. The next existence of the string can be substituted via a pointer to the earlier string in the form of pair.

## 4. Performance Validation

In this section, a detailed microarray image compression technique is provided. The proposed model is simulated using the MATLAB tool on a PC MSI Z370 A- Pro, i5-8600k, GeForce 1050Ti 4 GB, 16 GB RAM, 250 GB SSD, and 1 TB HDD. The parameter setting is given as follows: batch size: 500, number of epochs: 15, learning rate: 0.05, dropout rate: 0.25, and activation function: rectified linear unit (ReLU). The results are tested for five distinct images gathered from various sources.  Figure 3 illustrates some original and reconstructed images.

Table 1 provides an overall PSNR examination of the MRFOLBG-MIC model under five test images and distinct bit rates (BRs) [34].

Figure 4 demonstrates a brief comparative PSNR inspection of the MRFOLBG-MIC model under distinct BRs on image 1. The figure reported that the MRFOLBG-MIC model has offered improved PSNR values under all BRs. For instance, with a BR of 0.1875, the MRFOLBG-MIC method has offered a superior PSNR of 26.05 dB whereas the OLBGLZMA, CSALBG, FFA-LBG, HBMOLBG, QPSOLBG, and PSOLBG models have reached minimum PSNR of 24.79 dB, 23.59 dB, 21.83 dB, 21.02 dB, 20.13 dB, and 19.19 dB, respectively. Moreover, with a BR of 0.6250, the MRFOLBG-MIC technique has offered a higher PSNR of 34.53 dB whereas the OLBGLZMA, CSALBG, FFA-LBG, HBMOLBG, QPSOLBG, and PSOLBG models have reached lesser PSNR of 33.21 dB, 32.18 dB, 31.03 dB, 29.81 dB, 28.61 dB, and 27.40 dB correspondingly.

Figure 5 depicts a brief comparative PSNR analysis of the MRFOLBG-MIC model under distinct BRs in image 2. The figure reported that the MRFOLBG-MIC model has offered improved PSNR values under all BRs. For instance, with a BR of 0.1875, the MRFOLBG-MIC system has obtainable enhanced PSNR of 23.33 dB whereas the OLBGLZMA, CSALBG, FFA-LBG, HBMOLBG, QPSOLBG, and PSOLBG methods have obtained minimal PSNR of 21.69 dB, 20.23 dB, 19.19 dB, 17.70 dB, 16.40 dB, and 14.88 dB correspondingly. In addition, with a BR of 0.6250, the MRFOLBG-MIC method has accessible superior PSNR of 32.93 dB whereas the OLBGLZMA, CSALBG, FFA-LBG, HBMOLBG, QPSOLBG, and PSOLBG systems have achieved reduced PSNR of 31.77 dB, 30.59 dB, 28.93 dB, 27.20 dB, 25.94 dB, and 24.22 dB correspondingly.

Figure 6 showcases a brief comparative PSNR analysis of the MRFOLBG-MIC algorithm under distinct BRs on image 3. The figure exposed that the MRFOLBG-MIC model has offered improved PSNR values under all BRs. For instance, with a BR of 0.1875, the MRFOLBG-MIC model has presented a higher PSNR of 25.82 dB whereas the OLBGLZMA, CSALBG, FFA-LBG, HBMOLBG, QPSOLBG, and PSOLBG models have attained minimal PSNR of 24.71 dB, 23.47 dB, 22.66 dB, 20.88 dB, 19.31 dB, and 18.02 dB correspondingly. Furthermore, with a BR of 0.6250, the MRFOLBG-MIC method has offered a higher PSNR of 35.15 dB whereas the OLBGLZMA, CSALBG, FFA-LBG, HBMOLBG, QPSOLBG, and PSOLBG models have reached decreased PSNR of 33.66 dB, 31.94 dB, 30.28 dB, 28.99 dB, 27.73 dB, and 26.00 dB correspondingly.

Figure 7 portrays a brief comparative PSNR inspection of the MRFOLBG-MIC approach under distinct BRs in image 4. The figure outperformed that the MRFOLBG-MIC model has offered improved PSNR values under all BRs. For instance, with a BR of 0.1875, the MRFOLBG-MIC system has offered a superior PSNR of 25.49 dB whereas the OLBGLZMA, CSALBG, FFA-LBG, HBMOLBG, QPSOLBG, and PSOLBG methods have attained reduced PSNR of 24.03 dB, 22.45 dB, 21.22 dB, 20.22 dB, 19.12 dB, and 17.56 dB correspondingly. Eventually, with a BR of 0.6250, the MRFOLBG-MIC approach has offered a higher PSNR of 34.25 dB, whereas the OLBGLZMA, CSALBG, FFA-LBG, HBMOLBG, QPSOLBG, and PSOLBG models have gained minimal PSNR of 32.98 dB, 31.78 dB, 30.09 dB, 28.45 dB, 26.99 dB, and 25.64 dB, respectively.

Figure 8 exhibits a brief comparative PSNR analysis of the MRFOLBG-MIC method under distinct BRs on image 5. The figure reported that the MRFOLBG-MIC model has offered enhanced PSNR values under all BRs. For instance, with a BR of 0.1875, the MRFOLBG-MIC model has offered a higher PSNR of 24.81 dB whereas the OLBGLZMA, CSALBG, FFA-LBG, HBMOLBG, QPSOLBG, and PSOLBG models have attained decreased PSNR of 23.77 dB, 22.21 dB, 21.41 dB, 19.56 dB, 18.94 dB, and 16.87 dB, respectively. Followed by, with a BR of 0.6250, the MRFOLBG-MIC methodology has offered a higher PSNR of 34.71 dB whereas the OLBGLZMA, CSALBG, FFA-LBG, HBMOLBG, QPSOLBG, and PSOLBG models have reached decreased PSNR of 33.15 dB, 31.66 dB, 30.15 dB, 28.42 dB, 27.49 dB, and 26.06 dB correspondingly.

Figure 9 demonstrates a brief comparative PSNR inspection of the MRFOLBG-MIC technique under distinct BRs on image 6. The figure outperformed that the MRFOLBG-MIC model has offered improved PSNR values under all BRs. For instance, with a BR of 0.1875, the MRFOLBG-MIC method has offered a higher PSNR of 26.40 dB whereas the OLBGLZMA, CSALBG, FFA-LBG, HBMOLBG, QPSOLBG, and PSOLBG models have attained reduced PSNR of 25.08 dB, 23.16 dB, 22.07 dB, 20.33 dB, 20.03 dB, and 17.93 dB correspondingly. In addition, with a BR of 0.6250, the MRFOLBG-MIC model has offered a higher PSNR of 35.51 dB whereas the OLBGLZMA, CSALBG, FFA-LBG, HBMOLBG, QPSOLBG, and PSOLBG models have attained minimal PSNR of 34.72 dB, 32.86 dB, 31.39 dB, 28.97 dB, 28.94 dB, and 26.90 dB correspondingly.

In order to further ensure the improvements of the MRFOLBG-MIC technique, an average PSNR analysis is made in Table 2 and Figure 10. The results pointed out that the MRFOLBG-MIC model has resulted in increased values of average PSNR. For example with image 1, the MRFOLBG-MIC model has resulted in an increased average PSNR of 30.14 dB whereas the OLBGLZMA, CSALBG, FFALBG, HBMOLBG, QPSOLBG, and PSOLBG models have reached reduced average PSNR of 28.81 dB, 27.47 dB, 26.14 dB, 24.89 dB, 23.68 dB, and 22.42 dB, respectively. In addition, with image 6, the MRFOLBG-MIC model has resulted in an enhanced average PSNR of 31.61 dB whereas the OLBGLZMA, CSALBG, FFALBG, HBMOLBG, QPSOLBG, and PSOLBG techniques have reached lower average PSNR of 29.95 dB, 28.61 dB, 27.34 dB, 25.78 dB, 24.61 dB, and 23.20 dB correspondingly.

Finally, a comprehensive computation time (CT) inspection of the MRFOLBG-MIC model with other models is offered in Table 3 and Figure 11. From the figure, it is highlighted that the MRFOLBG-MIC model has resulted in reduced CT over the other models. For instance, with image 1, the MRFOLBG-MIC model has reached the least CT of 0.262s whereas the OLBGLZMA, CSALBG, FFALBG, HBMOLBG, QPSOLBG, and PSOLBG models have provided increased CT of 0.683s, 0.991s, 0.873s, 0.898s, 0.273s, and 0.263s, respectively. Also, with image 6, the MRFOLBG-MIC model has reached the least CT of 0.366s whereas the OLBGLZMA, CSALBG, FFALBG, HBMOLBG, QPSOLBG, and PSOLBG techniques have provided increased CT of 0.468s, 1.665s, 0.552s, 0.723s, 0.282s, and 0.362s correspondingly.

These results reported that the MRFOLBG-MIC model has shown effective compression efficiency over the other methods. The results indicated that the MRFOLBG-MIC model has accomplished enhanced performance due to the advantages of the MRFO algorithm.

## 5. Conclusion

In this study, a new MRFOLBF-MIC model has been presented to compress microarray images for effective storage and transmission. The LBG model is commonly utilized to design local optimal codebooks to compress images. The construction of codebooks can be defined as an NP hard problem and can be resolved by the MRFO algorithm. When the codebooks are produced by the MRFOLBG-MIC algorithm, Deflate model can be applied to compress the index tables, showing the novelty of the work. With a view to demonstrate the improved compression efficacy of the MRFOLBG-MIC model, a wide-ranging experimental validation process is performed using a benchmark dataset. The experimental outcomes inferred that the MRFOLBG-MIC model accomplished superior outcomes over the other existing models with an average PSNR of 31.61 dB and average CT of 0.262s. In future, compression then encryption schemes can be designed to securely transmit the microarray images in the real time environment. Besides, compression then encryption schemes can be designed to securely transmit the medial images.

## Figures and Tables

**Figure 1:** Steps in LBG.

**Figure 2:** Flowchart of MRFO.

**Figure 3:** Original images (first and third row) (second and fourth row).

**Figure 4:** PSNR analysis of MRFOLBG-MIC technique under image 1.

**Figure 5:** PSNR analysis of MRFOLBG-MIC technique under image 2.

**Figure 6:** PSNR analysis of MRFOLBG-MIC technique under image 3.

**Figure 7:** PSNR analysis of MRFOLBG-MIC technique under image 4.

**Figure 8:** PSNR analysis of MRFOLBG-MIC technique under image 5.

**Figure 9:** PSNR analysis of MRFOLBG-MIC technique under image 6.

**Figure 10:** Average PSNR analysis of MRFOLBG-MIC technique with existing approaches.

**Figure 11:** Average CT analysis of MRFOLBG-MIC technique existing methods.

**Algorithm 1:** Pseudocode of MRFO Algorithm.

**Table 1:** Overall PSNR analysis of the MRFOLBG-MIC technique under five test images and distinct BRs.

Test images	Methods	PSNR (dB)							
		0.1875	0.250	0.3125	0.3750	0.4375	0.500	0.5625	0.6250
*Image 1*	MRFOLBG-MIC	26.05	26.71	28.37	28.98	31.35	32.35	32.79	34.53
	OLBG-LZMA	24.79	25.65	27.15	27.98	29.62	30.59	31.50	33.21
	CSA-LBG	23.59	24.09	25.36	27.03	28.46	28.79	30.25	32.18
	FFA-LBG	21.83	23.17	23.84	25.58	27.59	27.32	28.74	31.03
	HBMO-LBG	21.02	21.70	22.38	23.98	26.48	26.18	27.57	29.81
	QPSO-LBG	20.13	20.49	21.42	22.32	25.55	24.66	26.24	28.61
	PSO-LBG	19.19	19.25	20.46	20.85	24.52	23.06	24.65	27.40

*Image 2*	MRFOLBG-MIC	23.33	23.95	25.46	27.45	28.48	30.16	31.26	32.93
	OLBG-LZMA	21.69	22.92	24.28	25.91	27.37	28.41	30.01	31.77
	CSA-LBG	20.23	21.19	22.90	24.80	25.88	27.57	28.85	30.59
	FFA-LBG	19.19	20.30	21.17	23.96	24.76	26.03	27.61	28.93
	HBMO-LBG	17.70	18.85	19.96	23.11	23.86	25.10	26.76	27.20
	QPSO-LBG	16.40	17.24	18.34	21.44	22.89	24.05	25.79	25.94
	PSO-LBG	14.88	15.97	17.41	20.60	22.07	23.04	24.73	24.22

*Image 3*	MRFOLBG-MIC	25.82	27.40	28.12	29.54	30.32	32.01	33.40	35.15
	OLBG-LZMA	24.71	25.63	26.48	28.13	29.08	30.73	32.00	33.66
	CSA-LBG	23.47	23.94	24.97	26.84	27.38	29.40	31.10	31.94
	FFA-LBG	22.66	23.06	23.97	25.20	26.23	27.86	30.06	30.28
	HBMO-LBG	20.88	21.74	22.54	24.02	25.06	26.58	28.54	28.99
	QPSO-LBG	19.31	20.24	21.41	23.04	24.24	25.76	27.44	27.73
	PSO-LBG	18.05	18.98	19.81	21.50	22.74	24.83	26.64	26.00

*Image 4*	MRFOLBG-MIC	25.49	26.98	28.46	30.00	31.44	32.38	33.07	34.25
	OLBG-LZMA	24.03	25.62	27.19	28.60	29.69	30.95	32.08	32.98
	CSA-LBG	22.45	24.70	25.89	27.06	28.52	29.64	30.43	31.78
	FFA-LBG	21.22	23.17	24.47	26.05	27.11	28.36	29.00	30.09
	HBMO-LBG	20.22	21.96	22.96	24.36	26.24	26.86	27.55	28.45
	QPSO-LBG	19.12	20.65	21.49	23.26	24.48	25.76	26.31	26.99
	PSO-LBG	17.56	19.04	19.75	22.04	23.43	24.36	24.60	25.64

*Image 5*	MRFOLBG-MIC	24.81	27.68	29.22	30.56	31.75	32.22	32.93	34.71
	OLBG-LZMA	23.77	26.07	27.36	27.93	29.09	30.75	31.61	33.15
	CSA-LBG	22.21	24.98	26.24	27.16	28.45	29.61	29.90	31.66
	FFA-LBG	21.41	23.24	24.82	26.23	26.92	28.32	29.79	30.15
	HBMO-LBG	19.56	22.27	23.58	24.34	27.04	26.49	26.93	28.42
	QPSO-LBG	18.94	20.66	21.08	23.08	24.24	26.31	26.23	27.49
	PSO-LBG	16.87	18.83	19.59	21.63	24.03	24.95	23.95	26.06

*Image 6*	MRFOLBG-MIC	26.40	28.71	29.75	31.82	33.33	33.12	34.27	35.51
	OLBG-LZMA	25.08	27.28	28.17	28.65	30.41	32.19	33.10	34.72
	CSA-LBG	23.16	25.80	27.34	28.42	29.49	30.37	31.43	32.86
	FFA-LBG	22.07	24.59	26.21	26.73	28.33	28.99	30.39	31.39
	HBMOLBG	20.33	23.09	24.30	25.83	27.85	27.94	27.89	28.97
	QPSO-LBG	20.03	22.20	22.35	24.13	25.05	26.99	27.18	28.94
	PSO-LBG	17.93	20.13	21.17	23.04	25.33	25.55	25.53	26.90

**Table 2:** Average PSNR analysis of MRFOLBG-MIC technique with existing approaches under various images.

Methods	Image 1	Image 2	Image 3	Image 4	Image 5	Image 6
MRFOLBG-MIC	30.14	27.88	30.22	30.26	30.49	31.61
OLBG-LZMA	28.81	26.55	28.80	28.89	28.72	29.95
CSA-LBG	27.47	25.25	27.38	27.56	27.53	28.61
FFA-LBG	26.14	23.99	26.17	26.18	26.36	27.34
HBMOLBG	24.89	22.82	24.79	24.83	24.83	25.78
QPSO-LBG	23.68	21.51	23.65	23.51	23.50	24.61
PSO-LBG	22.42	20.37	22.32	22.05	21.99	23.20

**Table 3:** Average CT analysis of MRFOLBG-MIC technique with existing approaches under various images.

Average Computation Time (sec)							
Methods	Image1	Image2	Image3	Image4	Image5	Image6	Average
MRFOLBG-MIC	0.262	0.318	0.266	0.281	0.328	0.366	0.304
OLBG-LZMA	0.683	0.548	0.425	0.588	0.552	0.468	0.544
CSA-LBG	0.991	1.431	1.068	1.675	1.683	1.665	1.419
FFA-LBG	0.873	0.707	0.667	0.647	0.646	0.552	0.682
HBMO-LBG	0.898	0.719	0.694	0.665	0.781	0.723	0.747
QPSO-LBG	0.273	0.337	0.344	0.270	0.250	0.282	0.293
PSO-LBG	0.263	0.341	0.263	0.269	0.310	0.362	0.301

## Data Availability

Data sharing is not applicable to this article as no datasets were generated during the current study.
